The article "EEG-Based Closed-Loop Neurofeedback for Attention Monitoring and Training in Young Adults" was published in 2021. Journal: J Healthc Eng.

# EEG-Based Closed-Loop Neurofeedback for Attention Monitoring and Training in Young Adults

**DOI:** 10.1155/2021/5535810

**Published:** 2021-06-14

**Authors:** Bingbing Wang, Zeju Xu, Tong Luo, Jiahui Pan

**Affiliations:** School of Software, South China Normal University, Guangzhou 510631, China

## Abstract

Attention is an important mechanism for young adults, whose lives largely involve interacting with media and performing technology multitasking. Nevertheless, the existing studies related to attention are characterized by low accuracy and poor attention levels in terms of attention monitoring and inefficiency during attention training. In this paper, we propose an improved random forest- (IRF-) algorithm-based attention monitoring and training method with closed-loop neurofeedback. For attention monitoring, an IRF classifier that uses grid search optimization and multiple cross-validation to improve monitoring accuracy and performance is utilized, and five attention levels are proposed. For attention training, we develop three training modes with neurofeedback corresponding to sustained attention, selective attention, and focus attention and apply a self-control method with four indicators to validate the resulting training effect. An offline experiment based on the Personal EEG Concentration Tasks dataset and an online experiment involving 10 young adults are conducted. The results show that our proposed IRF-algorithm-based attention monitoring approach achieves an average accuracy of 79.34%, thereby outperforming the current state-of-the-art algorithms. Furthermore, when excluding familiarity with the game environment, statistically significant performance improvements (*p* < 0.05) are achieved by the 10 young adults after attention training, which demonstrates the effectiveness of the proposed serious games. Our work involving the proposed method of attention monitoring and training proves to be reliable and efficient.

## 1. Introduction

Attention can be characterized as a cognitive process in the brain that selectively focuses on some part of the available information [1]. Nevertheless, excessive media multitasking poses a serious issue with respect to the attention function of young adults, resulting in distraction and poor attention control. Therefore, there is an increasing demand for attention monitoring and training for young adults [2].

Numerous methods have been developed for attention training, meditation [3], and computer-based exercises [4], but these approaches may contribute to mental fatigue. In recent years, several researchers have explored methods with fewer side effects. For example, Putri et al. [5] proposed the method of regular high-intensity circuit training (HICT), which can improve attention function in young male adults. In the same year, Luo and Zhang [2] conducted experiments to validate that noninvasive tactile training has an excellent effect on sustained attention in young adults. The main purpose of this paper is to investigate a method of attention monitoring and training based on closed-loop neurofeedback. We use brain-computer interface (BCI) technology, which utilizes recorded brain activity, primarily measured by electroencephalography (EEG), to execute communications between the brain and computers to manipulate the environment in a manner that is compatible with the intentions of humans [6]. Notably, EEG signals are the most frequently used. In contrast to the previously developed methods in [3, 4, 7], an EEG-based system can be used as a noninvasive neurofeedback platform to enhance individual attention and cognitive abilities [8]. Furthermore, a neurofeedback-based attention training system not only helps young adults but also is suitable for children, especially those with attention deficit hyperactivity disorder (ADHD) [9].

The article "EEG-Based Closed-Loop Neurofeedback for Attention Monitoring and Training in Young Adults" was published in 2021. Journal: J Healthc Eng.

BCI-based technology can be used to identify subtle shifts in individual attention [10]. Chiang et al. [11] developed an attention monitoring technique that integrates the minimum entropy principle approach (MEPA) and an associative Petri network (APN). Using a 14-electrode EEG device, a two-class classification accuracy of 90.4% was achieved based on 10 subjects in an online experiment. Hu et al. [12] compared the correlation-based feature selection (CFS) algorithm with other classification algorithms to evaluate attention at 3 levels (high, neutral, and low) and concluded that combining CFS and the K-nearest neighbors (KNN) data mining algorithm, which was used with a single valence resulted in the best performance. Six electrodes (C3, C4, Cz, P3, P4, and Pz) were used, and 10 subjects achieved an accuracy of 80.84% in their online experiment. In another study, Mohammadpour and Mozaffari [1] adopted an artificial neural network (ANN) to classify attention into four levels by using EEG signals from Fp1, Fp2, F3, F4, F7, F8, and Fz electrodes. An online experiment involving 5 subjects was conducted and an average accuracy of 79.75% was obtained. However, there have been two major issues to be further investigated. One issue is that the accuracy of attention monitoring needs to be improved, which may be related to the numbers of attention levels, detection algorithms, and types of feedback. The other issue is that more attention levels (i.e., ≥5) and fewer electrodes (i.e., ≤4) need to be explored in online attention monitoring, especially for EEG-based practical application.

The article "EEG-Based Closed-Loop Neurofeedback for Attention Monitoring and Training in Young Adults" was published in 2021. Journal: J Healthc Eng.

Neurofeedback is an effective training technique based on brain waves and computer processing [13], and EEG-based neurofeedback training can provide real-time information to individuals regarding their brain function through BCI devices. Bettencourt et al. [14] used closed-loop neurofeedback from multivariate pattern analysis (MVPA) as a type of cognitive prosthetic to provide a neural error signal so that individuals could learn to properly evaluate the state of their attention. Mohammadi et al. [13] designed a computer game to train individual attention based on neurofeedback, and they summarized that the neurofeedback game not only helps individuals increase the possibility of success in controlling their attention but also decreases the time required for the training process. Although EEG-based neurofeedback training plays an important role in attention improvement, one should note that the abovementioned training methods are not suitable for all the different mechanisms of attention, such as sustained attention, selective attention, and focus attention.

To address these above issues, we focus on EEG-based attention monitoring and training with closed-loop neurofeedback in this study. On one hand, we propose an improved random forest- (IRF-) algorithm-based monitoring method, which uses grid search optimization and multiple cross-validation to classify attention into five levels. The Personal EEG Concentration Tasks dataset involving 80 subjects was used to verify the effectiveness of the proposed attention monitoring method in the offline analysis. On the other hand, along with closed-loop neurofeedback, we provide three serious game-type training modes based on sustained attention, selective attention, and focus attention, which might be promising in terms of self-regulated attention training. Four primary indicators, including the Schulte times, win times, game scores, and skill times, were evaluated in an online experiment.

The rest of this paper is organized as follows: Section 2 offers additional details on various methods, such as EEG data processing, classification algorithms, and game design. The succeeding section illustrates the process of the experiments and analyzes the results, followed by a discussion and our conclusions.

## 2. Materials and Methods

This section provides an overview of the utilized methods, as shown in Figure 1, which are separated into two modules: EEG-based attention monitoring and EEG-based training. The first module commences with attention monitoring workflows based on EEG signals. Then, EEG data processing and feature extraction are performed. Finally, the output classification obtained based on the IRF algorithm is presented. In the second module, we illustrate the principle of attention training and describe the implementation of serious games with closed-loop neurofeedback.

The article "EEG-Based Closed-Loop Neurofeedback for Attention Monitoring and Training in Young Adults" was published in 2021. Journal: J Healthc Eng.

### 2.1. EEG-Based Attention Monitoring

In the attention monitoring module, an OpenBCI headset with 8 channels was used to collect EEG signals, and a wavelet transform algorithm was used to analyze and extract features for the preprocessed EEG data. Then, we utilized the IRF algorithm to classify attention.

#### 2.1.1. EEG Data Preprocessing and Feature Extraction

Previous related studies have shown that the power spectral densities (PSDs) of delta, theta, alpha, beta, and gamma have certain correlations with human attention. To this end, we selected and extracted EEG features based on these findings. An OpenBCI headset was used to capture the EEG data. Additionally, in terms of EEG data processing and attention monitoring, there are two factors to be considered. First, the most active sites of attention need to be given priority because the response is not evenly distributed across the electrodes. Second, if the algorithm is time-consuming, the time delays will not conform to the real-time constraints, rendering the feedback meaningless. Given the complexity of all kinds of data processing and the activity of positions, this paper selected the relatively active and attention-relative channels located in the frontal and temporal lobes, that is, TP9, AF7, AF8, and TP10, following the research of Castillo et al. [15] and Taillez et al. [16]. The wavelet transform algorithm was then applied to extract the PSD features of the EEG signals.

Wavelet analysis involves a combination of the time domain and frequency domain and is suitable for multiscale time-frequency analyses. The wavelet basis is defined as follows:

(1) $$\begin{array}{c} \psi_{s,a}\left(t\right)=\frac{1}{\sqrt{a}}\psi \left(\frac{t-s}{a}\right). \end{array}$$

In (1), *ψ*_*s*,*a*_(*t*) represents the displacement and scale expansion of the basic wavelet, which can be used to decompose signals at different times. *s* denotes the translation factor, *a* indicates the scale parameter, and $1/\sqrt{a}$ is the normalization factor, which is proportional to *ψ*_*s*,*a*_(*t*):

(2) $$\begin{array}{c} \text{CWT}\left(s,a\right)=\int_{-\infty }^{\infty }f\left(t\right)\psi_{s,a}\left(t\right)\text{d}t, \end{array}$$

(3) $$\begin{array}{c} f\left(t\right)=\frac{1}{C_{\psi }}\int \int_{-\infty +\infty }^{+\infty +\infty }\text{CWT}\left(s,a\right)\psi_{s,a}\left(t\right)\frac{\text{d}a\text{d}s}{\text{d}a^{2}}. \end{array}$$

In equation (2), a time-scale planar function CWT(*s*, *a*) mapped by the signal *f*(*t*) is shown. CWT(*s*, *a*) represents a one-dimensional continuous wavelet transform. *C*_*ψ*_=∫_−*∞*_^+*∞*^(|*ψ*(*u*)|^2^/|*u*|d*u*), and *ψ*(*u*) is the Fourier transform (FT) of *ψ*(*t*).

The article "EEG-Based Closed-Loop Neurofeedback for Attention Monitoring and Training in Young Adults" was published in 2021. Journal: J Healthc Eng.

The continuous wavelet transform (CWT) is used for extracting the PSD features of EEG signals. In this study, we used Daubechies coefficients for the wavelet transform, as they are characterized by excellent time localization performance and a maximal number of vanishing moments for a given support set. Daubechies 4 enjoys compact support and an orthonormal wavelet with smoothness. Thus, an improved effect can be achieved through the analysis of nonstationary EEG signals. It is necessary to select a suitable number of decomposition levels to analyze an EEG signal; thus, we selected a decomposition level of 5 (*L* = 5). In addition, the sampling frequency was 256 Hz, and the band-limited EEG was then subjected to a five-level decomposition coefficient of six subband signals through CWT. As shown in Figure 2, six subbands, including xD1, xD2, xD3, xD4, xD5, and xA1, represented the frequency range of the band-limited EEG signal [17], where xA is the decomposition approximation coefficient and xD is the decomposition detail coefficient.

Four wavelet thresholding methods were used in [18] to select an accurate threshold. We adopted the SURE threshold, which is an adaptive soft thresholding method. Once the threshold coefficients were extracted from each level, the effect of the noise on the EEG signals was removed. We then used the inverse CWT to reconstruct the signals at each level.

The first reconstructed detail D1 was regarded as the noise component of the EEG signal, and the reconstruction details of the other four subband signals D2–D5 and the reconstruction approximation of the subband signal A5 yielded signal information relevant to each EEG frequency band. Furthermore, 5 PSD features were extracted for classification: the delta (0 Hz < *f* < 4 Hz), theta (4 Hz < *f* < 8 Hz), alpha (8 Hz < *f* < 16 Hz), beta (16 Hz < *f* < 32 Hz), and gamma (32 Hz < *f* < 64 Hz) bands. There were a total of 20 EEG features (4 × 5 = 20).

#### 2.1.2. Improved Random Forest Classifier

Compared with the correlation classification method, random forest classification removes noise more effectively and accurately, which contributes to the higher accuracy during the classification of noise-containing EEG signals. In addition, the random forest method offers stability, running efficiency, and reducing errors for imbalanced datasets. On this foundation, Belle et al. [19] compared the random forest and regression techniques for attention classification based on EEG signals, determining that random forest seems to work best for both modalities, which obtained an average accuracy of 85.7% for EEG. Thus, we choose the random forest algorithm to classify the attention level and propose the IRF method with higher accuracy.

The article "EEG-Based Closed-Loop Neurofeedback for Attention Monitoring and Training in Young Adults" was published in 2021. Journal: J Healthc Eng.

The workflows of the IRF algorithm used for attention monitoring are shown in Figure 3. A random forest is a set of multiple decision tree classifiers {*h*(*x*, *ϕ*_*k*_), *k*=1,…}, and the parameter set {*ϕ*_*k*_} is an independent and identically distributed random vector. The input feature variables *X* are classified separately by each decision tree, and the results are relied on to make predictions. After that, the classification results with the most votes are attained as the output.

(1) *Decision Tree*. The random forest algorithm takes multiple samples from the original data through bootstrap resampling and generates multiple decision tree classification models. Three steps are involved in the establishment of a decision tree.

  Step 1. Select a random bootstrap sample across *N* original training sets by using the sampling with the replacement method, and repeat *k* times.
  Step 2. Train a decision tree with a training set including each bootstrap sample and recognize it as the root node of the sample. When each node is split, the feature variables *x*(*x* ≪ *X*) are extracted from the *X* total feature variables at random for calculation purposes, and the best feature obtained from the *x* feature variables is selected as a branch of the node to achieve minimal node impurity.
  Step 3. Split each node as before without a pruning operation in the course of establishing the decision tree.

To achieve stable accuracy, two random factors are introduced during the establishment of the decision tree. One is the bootstrap samples drawn from the *N* original training sets. The other is the stochastic feature variable selected from the node of the decision tree.

(2) *Voting*. To enhance the mutual influence between the classification models and improve their prediction ability, diverse decision trees are constructed by using different samples. After *k* rounds of training are conducted, the optimal classification models {*h*_1_(*X*), *h*_2_(*X*),…, *h*_*k*_(*X*)} are obtained and combined in a sequence to acquire the ultimate classification results by using the simple majority voting method. Equation (4) presents the classification decision:

(4) $$\begin{array}{c} H\left(x\right)=\arg\underset{Y}{\text{max}}\sum_{i=1}^{k}F\left(h_{i}\left(x\right)=Y\right), \end{array}$$

where *H*(*x*) is the classification model after the combination and *h*_*i*_(*x*) is one of the decision tree classification models. *Y* is the target variable, and the characteristic function is *F*(*h*_*i*_(*x*)=*Y*).

(3) *Grid Search Optimization*. The random forest algorithm has high precision and runs fast. However, a large number of hyperparameters are generated in the course of operation. To obtain attention monitoring results with high accuracy, a grid search is used to optimize the parameters. The grid search algorithm involves meshing the variable regions, traversing all the grid points, solving for the objective function values that satisfy the constraint conditions, and selecting the optimal values [20].  Figure 4 shows the workflow of the optimization process.

The article "EEG-Based Closed-Loop Neurofeedback for Attention Monitoring and Training in Young Adults" was published in 2021. Journal: J Healthc Eng.

To the best of our knowledge, it takes considerable time to traverse all the parameters, which decreases the training speed to some extent. In this paper, we use an improved grid search to increase the training speed. First, we use a large step size for a rough search over a wide range. The mesh built on the coordinate system consists of penalty parameters, the numbers of decision trees, and split features, n_estimators, max_features, and min_sample_leaf. When a set of parameters meets the set requirements, the optimal parameters and accuracy are output. In a case where more than one set of parameters meets the requirements, the set of parameters with the smallest penalty parameter is output as the best selection object. Then, the search range and step size are reduced to search the parameter set more accurately. The above steps are repeated with a step size of 2 to find the global hyperparameters.

(4) *Multiple Cross-Validation*. The accuracy of the proposed method is closely related to the ratio of training data to test data. To address this problem, *S*-fold cross-validation is conducted by randomly dividing the data into *S* subsets without repetition, of which *S* − 1 subsets are used for training and the remaining subset is used for testing:

(5) $$\begin{array}{c} \left\{T_{1},T_{2},\ldots ,T_{S}\right\},\\ \left(T_{i}\cap T_{j}=\emptyset \right). \end{array}$$

This process is repeated *S* times, and *S* accuracies are obtained. After each round, *S* − 1 subsets are selected at random to be retrained. In our paper, we use 10-fold cross-validation, which mitigates the situation of overfitting and yields reliable results. The training set is split into 10 subsets, of which one subset is used for testing and the remaining subsets are used as the training set.

### 2.2. Neurofeedback-Based Attention Training

Three types of attention mechanisms and closed-loop neurofeedback were adopted to implement the attention training function. Closed-loop neurofeedback technology involves the self-regulation of an individual's brain activity by relying on real-time visual and auditory feedback regarding his/her brain patterns. This technique can maintain specific conditions in the brain states of young adults and improve their cognitive function through training.

The article "EEG-Based Closed-Loop Neurofeedback for Attention Monitoring and Training in Young Adults" was published in 2021. Journal: J Healthc Eng.

We proposed an attention training method based on closed-loop neurofeedback technology that increases individual interest through the use of serious games and improves attention in a relaxing atmosphere without adverse reactions. At the same time, impaired concentration is associated not only with psychology but also with the three previously mentioned attention mechanisms: sustained attention, selective attention, and focus attention. According to the persistence, selectivity, and focus of attention, we designed three serious games (as shown in Figure 5), named Tug of War (Figure 5(a)), Adventures of Birds (Figure 5(b)), and Greedy Jelly (Figure 5(c)) in this study.

#### 2.2.1. Serious Games with Closed-Loop Neurofeedback

The young adults controlled each game by their attention levels; the specific implementation process is as follows: first, EEG signals were obtained from the young adults through OpenBCI. Then, their attention function was monitored by the IRF algorithm, and the results were quantified as young adults' attention levels during the games. The value of “high attention” was quantified as 1, the value of “medium-high attention” was quantified as 0.75, the value of “medium attention” was quantified as 0.5, the value of “medium-low attention” was quantified as 0.25, and the value of “low attention” was quantified as 0. In the sustained game, only when the young adults' attention levels were higher than a certain threshold would the strength of the character in the game be greater than that of the enemy. During the selective game, the bird's direction (upward, downward, or horizontal flight) was manipulated by the young adults' attention levels. For the focus game, the character, who was equipped with a special skill, would release his skill when the young adults' attention was focused and reached the maximum level. In Figure 5(d), a subject is shown playing a serious game with closed-loop neurofeedback.

To increase the efficiency of attention training, we optimized the graphical user interface (GUI) of the games as follows:

1. We designed various game environments and characters by taking young adults as the basis to increase their interest in the GUI.
2. Feedback was provided to the young adults in real time in the form of a progress bar that showed their attention levels.

Closed-loop neurofeedback technology can be an additional option for enhancing attention, which means that young adults could control the characters in the games with their attention; at the same time, they could also receive attention feedback from the games. Furthermore, young adults could increase their focus by actively concentrating after becoming acquainted with their attention function.

The article "EEG-Based Closed-Loop Neurofeedback for Attention Monitoring and Training in Young Adults" was published in 2021. Journal: J Healthc Eng.

## 3. Experiments and Results

### 3.1. Experiments for Attention Monitoring

#### 3.1.1. Offline Analysis

In offline analysis, the Personal EEG Concentration Tasks dataset involving 80 subjects was used to verify the effectiveness of the proposed attention monitoring method. We selected 70% of the samples as the training set and 30% of the samples as the test set at random. Different algorithms were utilized to divide attention into the abovementioned five levels. The results are shown in Table 1.

Among the five algorithms, the IRF achieved an accuracy of 79.34%, with a loss rate of 21.76%, a recall rate of 76.18%, and a precision of 82.60%. The results show that the attention monitoring method based on the IRF algorithm obtained the highest accuracy rate.

#### 3.1.2. Online Analysis

In the online experiment, we used an OpenBCI headset at 256 Hz to record the EEG data. Ten healthy subjects participated in the experiment, including 5 males and 5 females. The ages of the subjects ranged from 8 to 20 years old (mean = 15.95, std. = 4.63). The study was approved by the Ethics Committee of South China Normal University and complied with the Code of Ethics of the World Medical Association (Declaration of Helsinki). Before the experiment started, the subjects sat on a comfortable chair without blinking or moving their bodies, and they completed the entire experiment according to the provided instructions. There were two sessions during the experiment: a calibration session and an evaluation session.

In the calibration session, each subject performed 20 trials, which took the subjects approximately one hour to complete. Furthermore, each subject was asked to enter their personal information on a computer at the start of the experiment for the purpose of extracting the EEG data and labeling them conveniently. At the beginning of each trial, the computer screen showed a 10-second countdown to help subjects adjust their attention. After that, a calculation task, a minesweeping game task, or an article task was presented on the computer screen, and subjects needed to select an option or read. We induced the attention of subjects through the assigned task and recorded their EEG data simultaneously. After clicking the finish button, the subjects were asked to fill in the valence of self-assessment manikins (SAMs) to report their attention states, that is, high attention, medium-high attention, medium attention, medium-low attention, and low attention. The overall process of this experiment is illustrated in Figure 6.

The article "EEG-Based Closed-Loop Neurofeedback for Attention Monitoring and Training in Young Adults" was published in 2021. Journal: J Healthc Eng.

In the evaluation session, we used similar experimental trials to evaluate the model. In each trial, 6 algorithms (SVM, KNN, AdaBoost, ET, RF, and IRF) were applied to detect attention. Ultimately, we calculated the accuracy of each approach by comparing the predicted attention levels and the actual labels.

#### 3.1.3. Results

Figure 7 reveals the accuracy of the attention monitoring results for the 10 subjects, obtained by using the abovementioned five algorithms during the experiment. *P* values were calculated using a *t*-test to evaluate the accuracy differences between IRF and other algorithms with the SPSS tool, and the results are shown in Table 2, which were corrected for false discovery rate of *p* < 0.01.

The average accuracy rates of the various algorithms are displayed in Table 3, from which we can find that the accuracy of the IRF is significantly better than the accuracies of the other methods during the online attention monitoring experiment. There is a significant difference (*p*=0.016) between the IRF algorithm and ET algorithm.

### 3.2. Experiments for Attention Training

#### 3.2.1. Workflow of the Attention Training Experiment

Ten healthy subjects participated in this experiment, including 5 males and 5 females; these subjects were different from those who participated in the online experiment. The ages of the subjects ranged from 8 to 18 years (mean = 12.5, std. = 4.32). We performed a self-controlled study to validate the effectiveness of the training method, which offers good comparability and high reliability. During the course of the experiment, each subject sat quietly on a chair to avoid excessive movements that would affect the results.

Each subject performed 3 experiments. Before Experiment I and after each experiment, the subjects were required to complete a 5 × 5 grid of a Schulte table while recording the observed completion time and EEG signals.

There were 3 phases in each experiment: a preparation phase, a training phase, and a rest phase. The preparation phase, which lasted for 3 seconds, required subjects to actively refrain from noticing the game on the screen. During the training phase, the sustained game was presented, and the completion time was recorded. Afterwards, the selective game was carried out, and the scores were recorded when the subjects failed. Finally, the subjects performed the focus game and recorded the times at which they released the special skill. In addition, the resting phase provided a 5-second relaxation time during which subjects could divert their attention from the screen.

The article "EEG-Based Closed-Loop Neurofeedback for Attention Monitoring and Training in Young Adults" was published in 2021. Journal: J Healthc Eng.

#### 3.2.2. Effectiveness

Four primary indicators, including the Schulte times, win times, game scores, and skill times, are proposed as follows:

1. Schulte times, which represent the times(s) required to complete the Schulte table.
2. Win times, which denote the times(s) required to win a sustained game.
3. Game scores, which indicate the scores obtained by each subject upon losing the selective game.
4. Skill times, which denote the times at which the special skill was released during the focus game.

The Schulte times of the 10 subjects before Experiment I and after each experiment are shown in Figure 8. Figures 9(a)–9(c) show the win times, game scores, and skill times, respectively.

In the above four figures, all indicators underwent remarkable changes  (*p* < 0.05). The Schulte times and win times were obviously reduced. In contrast, the game scores and skill times increased significantly. These can be attributed to two reasons: (i) the familiarity of the subjects with the game environment after much practice and (ii) the effectiveness of neurofeedback. To explore the impact of the neurofeedback on the 3 experiments, we conducted an additional experiment without neurofeedback on the same subjects. We removed the neurofeedback elements from the three games in experiment III, such as the progress bar and the background sound effects used to display the subject's attention level in the GUI. The average results of the four indicators for each experiment are presented in Figure 10. For comparison purposes, we reduced the values of the win times by a factor of 10.

As the subjects became more familiar with the game, even without neurofeedback, their attention was improved to a certain extent. However, the rates of change of the four indicators without neurofeedback were much lower than those observed when using neurofeedback.

Moreover, to verify the accuracy of the control parameters, the Schulte times and the EEG signals input into the Schulte table before the experiment and after each experiment were analyzed. The Schulte times are often inversely proportional to the concentration and attention levels.  Table 4 illustrates the comparison between the Schulte times and the results of attention monitoring among the subjects. The results showed that the shorter a given Schulte time was, the more concentrated the subjects were and the higher the attention monitoring results. In contrast, there was less enhancement of the monitoring results.

## 4. Discussion

The main work in our paper was to propose an IRF-algorithm-based attention monitoring and training method with closed-loop neurofeedback. For attention monitoring, we divided attention into five levels ranging from low to high attention and applied the IRF algorithm to improve monitoring accuracy and performance. Furthermore, an offline experiment based on the Personal EEG Concentration Tasks dataset and an online experiment involving 10 young adults were carried out. The results yielded an average accuracy of 79.34% for the IRF algorithm. For attention training, we designed three training modes with neurofeedback, corresponding to sustained attention, selective attention, and focus attention. Furthermore, a self-control method with four indicators was used in the attention training experiment, and the results demonstrated a statistically significant performance improvement (*p* < 0.05) for the 10 tested young adults after attention training, thereby demonstrating the effectiveness of the proposed games.

The article "EEG-Based Closed-Loop Neurofeedback for Attention Monitoring and Training in Young Adults" was published in 2021. Journal: J Healthc Eng.

From the perspective of the attention monitoring method, it is essential to achieve a promising level of accuracy and improved classification. At the same time, the attention mechanism and training method are vital for attention training. We show the differences between other studies and our work in Tables 5 and 6.

Most past studies explored attention training methods, such as the focused attention meditation (FAM) method proposed by Yoshida et al. [24]. In addition, Shereena et al. [25] used the EEG neurofeedback training method to design training tasks, aiming to enhance *β* waves for the purpose of suppressing *θ* waves. These studies related to attention training focused on EEG signals, with little emphasis on neurofeedback. Notably, several recent papers examined the method of combining neurofeedback and serious games, which is helpful for improving self-regulation skills in attention training with appropriate guidance; an example of this is the “ExerBrain” game [14], which assists individuals in improving their attention control due to the immersive and interactive feature of neurofeedback. Moreover, neurofeedback training has proven to be an efficient tool for sustained attention [26]. Nevertheless, attention, as a kind of higher-order cognition, comprises not only sustained attention but also selective attention and focus attention [25]. As such, this study provides a means by which to implement serious games and analyze three mechanisms of attention simultaneously to help young adults enhance their attention effectively.

The advantages of this paper primarily comprise the following points: (i) we utilized the IRF algorithm for five-level attention monitoring and obtained promising accuracy; (ii) we designed serious games in a multiangle and targeted manner with consideration of sustained, selective, and focus attention; (iii) we quantified the attention monitoring results and used them as the control parameters to manipulate the games with improved accuracy; and (iv) four indicators were proposed in the experiment to validate the effectiveness of the presented method.

The article "EEG-Based Closed-Loop Neurofeedback for Attention Monitoring and Training in Young Adults" was published in 2021. Journal: J Healthc Eng.

In addition, the main finding is that the attention of young adults could be enhanced by using closed-loop neurofeedback in comparison with methods that ignore neurofeedback. This is in line with the results of previous attention monitoring studies [27]. On this basis, this paper used the IRF algorithm to classify 5-level attention and attained an accuracy of 79.34%, which is higher than those of the other algorithms that were compared. Furthermore, consistent with past studies [11, 25], we showed that neurofeedback training can assist young adults in improving their attention. In the present study, we implemented three serious games for young adults with neurofeedback and incorporated three mechanisms of attention that were not fully considered in past studies. Furthermore, the attention training method in this paper contributed to significant improvements in sustained attention, selective attention, and focus attention. Therefore, we can conclude that all mechanisms of attention can be improved with specific serious games.

The primary limitation of our study was the small number of subjects examined during the experiment. In addition, there are a few datasets pertaining to the attention of young adults; these data are challenging to record due to the volatility of conductive media in BCIs. In addition, several external factors, such as the habits, motivations, and mental statuses of the subjects, were not considered.

## 5. Conclusions

We proposed an IRF-algorithm-based attention monitoring and training method with closed-loop neurofeedback, and we presented the mechanism of attention. In the future, we will collect attention data and attempt to fuse EEG and physiological signals (such as facial expressions and verbal speech) to improve the accuracy of attention monitoring. Furthermore, we will develop 3D serious games in the near future.

## Figures and Tables

**Figure 1:** Architecture of the attention monitoring and training modules.

**Figure 2:** Wavelet multiresolution analysis.

**Figure 3:** Workflows of the improved random forest algorithm used in attention monitoring.

**Figure 4:** Workflow of the optimization process.

**Figure 5:** Three serious games were developed to improve attention. (a) Tug of War was designed in terms of the mechanism of sustained attention. (b) Adventures of Birds was designed in terms of the mechanism of selective attention. (c) Greedy Jelly was designed in terms of the mechanism of focus attention. (d) A subject playing a serious game with closed-loop neurofeedback.

The article "EEG-Based Closed-Loop Neurofeedback for Attention Monitoring and Training in Young Adults" was published in 2021. Journal: J Healthc Eng.

**Figure 6:** Workflow of the attention monitoring experiment.

**Figure 7:** Accuracies (%) of the five-level attention results obtained via the SVM, KNN, AdaBoost, ET, RF, and IRF algorithms in online experiments. The *x*-axis of each subfigure corresponds to the subject IDs, and the *y*-axis corresponds to the accuracy rates (%).

**Figure 8:** Schulte times before the experiment and during experiment (I), experiment II, and experiment III. The *x*-axis of each subfigure corresponds to the subject IDs, and the *y*-axis corresponds to the Schulte times.

**Figure 9:** The win times (a), game scores (b), and skill times (c) obtained during experiment (I), experiment II, and experiment III. The *x*-axis of each subfigure corresponds to the subject IDs, and the *y*-axis corresponds to the performances of the corresponding indicators.

**Figure 10:** Average results of the four indicators in experiment (I), experiment II, and experiment III. The *x*-axis of each subfigure identifies each indicator, and the *y*-axis corresponds to the Schulte times, one-tenth of the win times, the game scores, and the skill times.

**Table 1:** Accuracy (%) of five-level attention monitoring with different algorithms.

Algorithm	Accuracy	Loss	Recall	Precision
Support vector machine (SVM)	52.46	51.48	26.65	53.41
K-nearest neighbors (KNN)	54.75	43.60	50.81	50.12
AdaBoost	67.32	32.35	68.74	71.69
Extreme random tree (ET)	72.90	27.28	65.68	81.09
Random forest (RF)	73.22	26.45	64.02	79.54
Improved random forest (IRF)	79.34	21.76	76.18	82.60

**Table 2:** Results of a *t*-test with SPSS.

Group	SVM-IRF	KNN-IRF	AdaBoost-IRF	ET-IRF	RF-IRF
*t*-test statistics	−29.347	−30.623	−9.565	−7.753	−20.622
*P* value	<0.001	<0.001	<0.001	<0.001	<0.001

**Table 3:** Average accuracy rates (%) of various algorithms for five levels of attention in online experiments.

Algorithm	SVM	KNN	AdaBoost	ET	RF	IRF
Accuracy (%)	48.52 ± 5.35	50.49 ± 4.26	62.62 ± 4.70	72.95 ± 5.38	73.14 ± 5.93	79.06 ± 6.47

**Table 4:** Comparison of the Schulte times and the results of attention monitoring.

Subject	Before the experiment		Experiment I		Experiment II		Experiment III	
	*T*	*D*	*T*	*D*	*T*	*D*	*T*	*D*
1	25.12	Medium-low	16	High	15	High	14	High
2	34	Low	30	Low	26.8	Low	25	Medium-low
3	21.1	Medium	18.37	Medium-high	15.64	High	12.91	High
4	20.55	Medium-high	19.17	Medium-high	19	Medium-high	17	High
5	23.3	Medium-	19.25	Medium-high	18	Medium-high	16	High
6	32.07	Low	29	Low	28	Low	22	Medium
7	24.35	Medium-low	20.05	Medium-high	18	Medium-high	17.5	High
8	20.37	Medium-high	16.32	High	16	High	15.6	High
9	21.25	Medium	21	Medium	20	Medium-high	18	Medium-high
10	26	Medium-low	24.5	Medium-low	22	Medium	20	Medium-high

*Note*. *T* denotes the Schulte time of each subject, and *D* denotes the monitoring result of each subject.

The article "EEG-Based Closed-Loop Neurofeedback for Attention Monitoring and Training in Young Adults" was published in 2021. Journal: J Healthc Eng.

**Table 5:** Comparison of different methods related to attention monitoring.

Reference	Algorithm	Classification	Accuracy (%)
[1]	ANN	4 levels	78
[21]	KNN	3 levels	67
[22]	Naive Bayes	3 levels	60
Our work	IRF	5 levels	79.34

**Table 6:** Comparison of different methods related to attention training.

References	Mechanism	Method
[2]	Sustained attention	A closed-loop tactile training process related to visual sustained attention.
[14]	Sustained attention	Closed-loop neurofeedback from MVPA as a type of cognitive prosthetic.
[23]	Sustained attention and selective attention	A 3D game with neurofeedback.
Our work	Sustained attention, selective attention, and focus attention	Three serious games related to the mechanism of attention with neurofeedback.

## Data Availability

All the data included in this study are available upon request by contacting the corresponding author.

## References

[1] Mohammadpour M., Mozaffari S. Classification of EEG-based attention for brain computer interface.

[2] Luo Y., Zhang J. (2020). The effect of tactile training on sustained attention in young adults. *Brain Sciences*.

[3] Chen R., Yang Z., Li J. (2020). State and short-term effects of mindfulness meditation training on attention. *Journal of Vision*.

[4] Tang Y.-Y., Posner M. I. (2009). Attention training and attention state training. *Trends in Cognitive Sciences*.

[5] Putri T. A., Muniroh M., Purwoko Y. (2020). Regular high intensity circuit training improves attention function and reaction time among male young adults. *Malaysian Journal of Medicine and Health Sciences*.

[6] Abiri R., Borhani S., Sellers E. W., Jiang Y., Zhao X. (2019). A comprehensive review of EEG-based brain-computer interface paradigms. *Journal of Neural Engineering*.

[7] Liu M., Zhang J., Jia W. (2019). Enhanced executive attention efficiency after adaptive force control training: behavioural and physiological results. *Behavioural Brain Research*.

[8] Belkacem A. N., Jamil N., Palmer J. A., Ouhbi S., Chen C. (2020). Brain computer interfaces for improving the quality of life of older adults and elderly patients. *Frontiers in Neuroscience*.

[9] Qian X., Loo B. R. Y., Castellanos F. X. (2018). Brain-computer-interface-based intervention re-normalizes brain functional network topology in children with attention deficit/hyperactivity disorder. *Translational Psychiatry*.

[10] Kosmyna N., Maes P. (2019). AttentivU: an EEG-based closed-loop biofeedback system for real-time monitoring and improvement of engagement for personalized learning. *Sensors*.

The article "EEG-Based Closed-Loop Neurofeedback for Attention Monitoring and Training in Young Adults" was published in 2021. Journal: J Healthc Eng.

[11] Chiang H.-S., Hsiao K.-L., Liu L.-C. (2018). EEG-based detection model for evaluating and improving learning attention. *Journal of Medical and Biological Engineering*.

[12] Hu B., Li X., Sun S., Ratcliffe M. (2018). Attention recognition in EEG-based affective learning research using CFS+KNN algorithm. *IEEE/ACM Transactions on Computational Biology and Bioinformatics*.

[13] Mohammadi H. S., Pirbabaei E., Sisi M. J., Sekhavat Y. A. ExerBrain: a comparison of positive and negative reinforcement in attention training using BCI based computer games.

[14] Bettencourt M. T., Cohen J. D., Lee R. F. (2015). Closed-loop training of attention with real-time brain imaging. *Nature Neuroscience*.

[15] Castillo O., Sotomayor S., Kemper G., Clement V. Correspondence between TOVA test results and characteristics of EEG signals acquired through the muse sensor in positions AF7-AF8.

[16] Taillez T., Kollmeier B., Meyer B. T. (2020). Machine learning for decoding listeners’ attention from electroencephalography evoked by continuous speech. *European Journal of Neuroscience*.

[17] Al-Qazzaz N., Hamid Bin Mohd Ali S., Ahmad S., Islam M., Escudero J. (2015). Selection of mother wavelet functions for multi-channel EEG signal analysis during a working memory task. *Sensors*.

[18] Al-Qazzaz N. K., Ali S., Ahmad S. A., Islam M. S., Ariff M. I. Selection of mother wavelets thresholding methods in denoising multi-channel EEG signals during working memory task.

[19] Belle A., Hargraves R. H., Najarian K. (2012). An automated optimal engagement and attention detection system using electrocardiogram. *Computational and Mathematical Methods in Medicine*.

[20] Wang X., Gong G., Li N., Qiu S. (2019). Detection analysis of epileptic EEG using a novel random forest model combined with grid search optimization. *Frontiers in Human Neuroscience*.

[21] Li Y., Li X., Ratcliffe M. A real-time EEG-based BCI system for attention recognition in ubiquitous environment.

[22] Srinivasan R., Thorpe S., Deng S., Lappas T., D’Zmura M. Decoding attentional orientation from EEG spectra.

[23] Thomas K. P., Vinod A. P., Cuntai Guan C. Design of an online EEG based neurofeedback game for enhancing attention and memory.

[24] Yoshida K., Takeda K., Kasai T. (2020). Focused attention meditation training modifies neural activity and attention: longitudinal EEG data in non-meditators. *Social Cognitive and Affective Neuroscience*.

[25] Shereena E. A., Gupta R. K., Bennett C. N., Sagar K. J. V., Rajeswaran J. (2019). EEG neurofeedback training in children with attention deficit/hyperactivity disorder: a cognitive and behavioral outcome study. *Clinical EEG and Neuroscience*.

The article "EEG-Based Closed-Loop Neurofeedback for Attention Monitoring and Training in Young Adults" was published in 2021. Journal: J Healthc Eng.

[26] Jirayucharoensak S., Israsena P., Pan-Ngum S., Hemrungrojn S., Maes M. (2019). A game-based neurofeedback training system to enhance cognitive performance in healthy elderly subjects and in patients with amnestic mild cognitive impairment. *Clinical Interventions in Aging*.

[27] Kosmyna N., Morris C., Sarawgi U. Attentivu: a biofeedback system for real-time monitoring and improvement of engagement.

